# The Effect of Preoperative Rehabilitation Training on the Early Recovery of Joint Function after Artificial Total Knee Arthroplasty and Its Effect Evaluation

**DOI:** 10.1155/2022/3860991

**Published:** 2022-01-25

**Authors:** Yuliu Zheng, Zida Huang, Liqun Dai, Yu Liu, Yanqin Chen, Wenming Zhang, Rongjin Lin

**Affiliations:** ^1^The First Afilliated Hospital of Fujian Medical University, Fuzhou 350004, China; ^2^The First Clinical Medical College of Fujian Medical University, Fuzhou 350004, China

## Abstract

**Objective:**

To study the effect of preoperative rehabilitation training on the rehabilitation of patients after total knee arthroplasty.

**Methods:**

A total of 120 patients diagnosed with knee osteoarthritis and undergoing total knee arthroplasty were selected and divided into experimental group and control group according to a random number table, with 60 cases in each group. The control group only carried out routine clinical nursing before the operation, and the experimental group used the formulated preoperative rehabilitation training method based on the control group for training. By comparing the visual analogue score (VAS), keen society score (KSS), postoperative time to get out of bed for the first time, patient satisfaction, and other related indicators between the two groups of patients, the recovery of keen joint function of patients after surgery was evaluated.

**Results:**

The visual analogue scale (VAS) of the experimental group was significantly lower than that of the experimental group at three days after operation. The keen society score (KSS) of the experimental group was significantly better than that of the control group at three days after surgery and one month after surgery. The time to get out of bed for the first time after operation in the experimental group (44.93 ± 13.63) was significantly less than that in the control group (78.33 ± 13.52). The patient satisfaction of the experimental group was significantly higher than that of the control group (88.30 ± 3.61). The above statistical results were all *p* < 0.05 of the two groups, and the differences were statistically significant.

**Conclusion:**

Preoperative rehabilitation training can significantly reduce the pain of patients after knee replacement, improve the functional state of knee joints, shorten the time to get out of bed for the first time after surgery, and win the best recovery opportunity, which can better improve patient satisfaction in hospitalization and improve medical care services level.

## 1. Introduction

Knee arthroplasty (TKA), also known as total knee resurfacing, is an effective treatment for end-stage knee joint diseases (such as osteoarthritis and rheumatoid arthritis). Surgery replaces the weight-bearing surface of the knee joint with artificial implants to reduce pain and improve mobility [1]. In recent years, the number of global TKA surgeries has continued to increase [2]. China is the country with the largest elderly population in the world, accounting for one-fifth of the global elderly population, and it is the country with the fastest aging rate [3]. Although total knee arthroplasty (TKA) is the most important and effective method to relieve pain and improve functional recovery [4], doctors are worried about the pain and functional recovery of patients after surgery [5–7]. Literature studies indicate that 30% of patients still have varying degrees of pain after TKA surgery [8], and knee joint function has not been well recovered [9]. Many literature studies have also been done on the effects of preoperative functional exercises on knee joint function, but most of them are 6–8 weeks before surgery or even three months before surgery [10, 11]. According to reports, preoperative training plan has an effect on enhancing the strength of the quadriceps, which helps to promote postoperative functional recovery and relieve pain [12, 13]. Some reports have found that there is no beneficial effect on postoperative functional recovery [14]. Based on the above literature review, there is no investigation and research on the preoperative functional exercises performed on patients 3 days before surgery. Combined with the current situation of our department, it is planned to conduct preoperative rehabilitation training for patients who will undergo TKA surgery 3 days before surgery to ensure patients receive designated training before surgery to improve their compliance with postoperative rehabilitation and improve their self-confidence, thereby reducing the patient's early pain and maximizing early joint function recovery. The theory of prehabilitation was first proposed by Ditmyer and applied to orthopedic perioperative rehabilitation. Its content covers rehabilitation assessment, rehabilitation treatment, and rehabilitation education. It is recommended to optimize the joint function of patients through exercise before surgery [15, 16]. With the advancement of the concept of accelerated rehabilitation, preoperative rehabilitation training is a trend, and preoperative prerehabilitation programs with exercise as the core become more important. This study aims to explore the application and impact analysis of preoperative rehabilitation training after total knee arthroplasty.

## 2. Materials and Methods

### 2.1. General Information

This study adopted a convenient sampling method and selected 120 patients who underwent total knee arthroplasty in tertiary class A in Fujian province from 2019.09.19 to 2021.03.19. This study was approved by the Ethics Committee of the First Affiliated Hospital of Fujian Medical University. The batch number is No. 252, No. 1. Among them, there were 60 cases in the observation group, 8 males and 52 females, aged 66.97 ± 9.04; 60 cases in the experimental group, 18 males and 42 females, aged 67.33 ± 7.91. In total, there were 26 males and 94 females. The male-to-female ratio was 1 : 3.6 times. Inclusion criteria were as follows: ① patients who can actively cooperate; ② preoperatively diagnosed as knee osteoarthritis or rheumatoid arthritis; ③ receiving unilateral total knee arthroplasty; ④ clear consciousness, normal communication skills, and no cognition and communication barriers; ⑤ informed and agreed to participate in this research. Exclusion criteria were as follows: ① patients with knee arthritis caused by other diseases, such as rheumatoid arthritis; ② patients who have undergone other joint replacement surgeries; ③ patients with bilateral total knee replacement surgery; ④ patients with severe postoperative complications.; ⑤ patients with multiple organ failure and other patients that affect the quality of life.

### 2.2. Method

#### 2.2.1. Intervention Methods

This group of research is divided into the observation group and experimental group. Unilateral total knee arthroplasty is performed in our department. The experimental group adopted the pre rehabilitation training method [17]: the pre-rehabilitation training method mainly refers to the training materials for residents of rehabilitation medicine and the accelerated rehabilitation and perioperative management of modern joint replacement (1) Ankle pump training: when performing ankle joint activities, try to make the ankle joint reach the maximum angle as much as possible, maintain it for 5 s, and relax for 5 s, 20 times/group, 10 groups/d; (2) quadriceps isometric contraction training: the patient lies flat on the bed, raises the back of the ankle joint, tightens the anterior thigh muscles, keeps the patella fixed, maintains for 5 s, and relaxes for 5 s, 20 times/group, 4–6 groups/d; (3) straight leg raising training: straighten the knee joint as much as possible and lift it 20 cm away from the bed surface, maintain it for 15 s, and then put it back in place, 20 times/group, with an interval of 5 s each time, 4–6 groups/d; (4) knee joint active flexion and extension training (AROM): the patient takes a sitting position, flexes the knee joint to the maximum angle, maintains it for 5 seconds, then tries their best to straighten the knee joint, maintains it for 5 seconds, and returns to the original position, 20 times/group, 4–6 groups/d; (5) knee joint passive flexion and extension training (PROM): the patient takes a sitting position, presses down the affected leg with the uninvolved leg to increase the flexion angle, maintains it for 5 seconds, and restores the original position, 20 times/group, 4–6 groups/d; (6) hamstring contraction training: the patient takes a standing position, raises the calf backwards to the maximum angle, persists for 20 s, and returns to the original position, 20 times/group, each interval is 5 s, 4–6 groups/d; (7) in situ stepping training: maintain body balance and correct abnormal gait in time, 2 minutes/time, 10 times/d; (8) stand up from bed and gait exercise: teach patients to master the use of walkers. Ankle pump training and quadriceps muscle contraction training were started within 12 hours after the operation. After 24 hours, the above 8 exercises were trained in sequence. The observation group did not take preoperative rehabilitation training before surgery and started ankle pump training and quadriceps contraction training within 12 hours after surgery.

#### 2.2.2. Evaluation Index

1. At present, there is no unified standard for “early getting out of bed” after joint replacement at home and abroad. This study uses the time to get out of bed for the first time after the operation as the evaluation standard; that is, the patient feels good after the operation, and it is based on standing or walking for the first time [18].
2. Using the visual analogue scale (VAS) of pain, the patients will score according to their own pain level. The score is 0–10 points. The higher the score, the more severe the pain.
3. Keen society score: pain (50 points), stability (25 points) and mobility (25 points); total clinical score: 100 points; excellent: 85 ∼ 100 points; good: 70 ∼ 84 points; fair: 60 ∼ 69 points; poor: < 60 points.
4. Statistical methods are based on the clinical data of the two groups. Software used for the analysis is R version 4.0.3. The measurement data are described by the mean ± standard deviation. The difference between the groups is compared with two independent samples. The *t*-test is used for the count data. The number of cases (percentage) was described, and the difference between groups was compared by chi-square test. The paired *t*-test was used to compare the pain scores one day after the operation and three days after the operation. The KSSs were compared using repeated measures analysis of variance with one of the two factors being repeated measures. Inspection level *α* = 0.05, two-sided inspection.

## 3. Results

The difference between the experimental group and the control group in age, complications, length of stay before surgery, infection, total hospitalization cost, hemoglobin, and albumin is not statistically significant (all *p* > 0.05), and it is comparable; see Table 1.

There were significant differences between the experimental group and the observation group in the first time (*H*), pain, and satisfaction (*p* < 0.05) after operation, as shown in Table 2.

The difference of 3-day pain between different groups was statistically significant (*t* = 4.796, *pt* = 0.001), and the pain score (1.22 ± 0.67) of the experimental group was significantly lower than that of the observation group (1.83 ± 0.74) (*p* < 0.05); see Table 3.

Comparisons between groups at the same time point are illustrated as follows: there was no significant difference between the control and experimental groups in preoperative KSSs (*F* = 0.000, *p* = 0.988 > 0.05), and the control and experimental patients were comparable in preoperative KSSs. There was no significant difference in KSSs between the two groups at 1 day after surgery (*F* = 0.667, *p* = 0.416 > 0.05). The KSSs at 3 days and 1 month were significantly different between the two groups (*F* = 68.734, *p* < 0.001), (*F* = 111.462, *p* < 0.001). The KSSs of the control group were significantly lower than those of the experimental group, and it can be seen that from the third postoperative day, preoperative rehabilitation training was significantly better than the control group in improving the knee function of patients after knee arthroplasty (Table 4).

## 4. Discussion

1. Osteoarthritis (knee osteoarthritis) of the knee joint (KOA) is one of the most common diseases of the elderly in China, among >60-year-olds, the incidence is about 15.7%, the ratio of men to women is approximately 1 : 2, and the incidence increases with age [19]. The ratio of men to women in this study was 1 : 3.6. Epidemiological surveys show a ratio of 1 : 3.72 [20]. Data research shows that women should strengthen knee management, exercise and protect their joints appropriately, learn knee nursing knowledge, and prevent chronic knee injury.
2. Hamada D and other studies show that total knee arthroplasty can effectively correct knee deformities, relieve knee pain, and improve knee function, but its preoperative and postoperative rehabilitation function training directly affect the [21] effect of surgery and recovery. Through the analysis of Table 2, it can be seen that the first time (*H*), pain, and satisfaction (score) of the experimental group after operation were significantly higher than those of the observation group (*p* < 0.05). It can be seen that the effect of precomfort training on patients is significant and meaningful. Studies have shown that the specific and quantitative content of rehabilitation training can enhance the time of bedside communication, actively guide patients to carry out early active training, and urge patients to complete rehabilitation exercise content daily so that patients from passive treatment to active participation in treatment effectively improve self-management ability and rehabilitation training compliance [22]. The results of this study show that preoperative rehabilitation training can effectively enhance the ability of patients to get out of bed, improve the ability of autonomous exercise rehabilitation, reduce postoperative pain, and improve the clinical satisfaction of patients.
3. Preoperative rehabilitation is a preoperative exercise-centered regimen that improves patients' function, optimizes their physiological reserves, and adapts them to withstand surgical stress so that their postoperative functional status can be restored to preoperative and daily life faster [23]. In this study, there was no significant difference in pain between the two groups before operation and 1 day after operation. The pain score of the experimental group was significantly lower than that of the observation group 3 days after operation. It can be seen that preoperative rehabilitation training can enhance the muscle strength of the patients, increase the tolerance of pain, and obviously alleviate postoperative pain under the same conditions. Previous studies have shown that patients will have pain and swelling due to joint fixation and peripheral tissue debridement. Severe pain will limit the patient's active and passive activities, which is an important factor affecting the patient's enthusiasm for postoperative functional training and the degree of knee stiffness [24]. It can be seen that rehabilitation training intervention is particularly important after knee arthroplasty.
4. Knee arthroplasty is the main method for clinical treatment of various knee diseases. However, there are problems such as prolonging the recovery time of patients' joint function, limiting patients' activities, causing unstable emotions such as anxiety, depression, and fear, and reducing patients' compliance with rehabilitation training [25]. Research shows that there were 40–65% of patients who did not insist on rehabilitation exercise [26] after knee arthroplasty. This study shows that the planned preoperative rehabilitation training in the experimental group can promote the rehabilitation in a short time. That is to restore patients' confidence, alleviate patients' concerns, and increase patients' trust in medical personnel. As the operation lasted longer, knee function improved. One month after operation, the knee function was 91.97 ± 2.31. Although the observation group did not conduct preoperative rehabilitation training, the knee function also increased with the duration of surgery. One month after operation, the knee function was 87.40 ± 2.43. The knee function of the experimental group and the observation group was significantly improved before operation and 1 day, 3 days, and 1 month after operation.

## 5. Summary

Knee arthroplasty is an effective measure to improve knee pain and knee dysfunction in elderly patients. Therefore, the planned prerehabilitation training before operation is beneficial to the high quality of knee joint function, which solves the problem that patients miss the best rehabilitation opportunity because of the lack of exercise and ensures the maximum rehabilitation of joint function.

## Figures and Tables

**Table 1:** Analysis of the basic information included in the study.

	Total (*n* = 120)	Observation group (*n* = 60)	Experimental group (*n* = 60)	*t*/*x*^*2*^	*p*
Gender				4.910	0.027
Male	26 (21.67)	8 (13.33)	18 (30.00)		
Female	94 (78.33)	52 (86.67)	42 (70.00)		
Age	67.15 ± 8.46	66.97 ± 9.04	67.33 ± 7.91	−0.236	0.814
Complications				0.988	0.320
No	111 (95.69)	59 (98.33)	52 (92.86)		
Yes	5 (4.31)	1 (1.67)	4 (7.14)		
Preoperative hospitalization days	2.98 ± 2.09	2.83 ± 1.45	3.14 ± 2.59	−0.793	0.429
Infection				0.000	1.000
Yes	2 (1.67)	1 (1.67)	1 (1.67)		
No	118 (98.33)	59 (98.33)	59 (98.33)		
Total hospitalization costs	52494.59 ± 10913.44	52470.10 ± 10294.62	52519.08 ± 11586.40	−0.024	0.981
Hemoglobin	112.11 ± 13.99	111.90 ± 14.20	112.32 ± 13.90	−0.162	0.871
Albumin	36.34 ± 3.43	36.70 ± 3.38	35.98 ± 3.47	1.162	0.247

**Table 2:** Statistical analysis of the indicators of the study.

	Total (*n* = 120)	Observation group (*n* = 60)	Experimental group (*n* = 60)	*t/x* ^*2*^	*p*
Getting out of bed for the first time after operation	61.63 ± 21.54	78.33 ± 13.52	44.93 ± 13.63	13.477	<0.001
Pain 1 day after operation	3.82 ± 0.90	3.88 ± 0.90	3.75 ± 0.89	0.812	0.418
Pain after 3 days	1.52 ± 0.77	1.83 ± 0.74	1.22 ± 0.67	4.796	<0.001
Satisfaction (score)	90.40 ± 4.22	88.30 ± 3.61	92.50 ± 3.73	−6.264	<0.001
Hospitalization days	8.66 ± 3.13	8.38 ± 2.62	8.93 ± 3.57	−0.961	0.339
Therapeutic effects				0.076	0.783
Improvement	15 (12.50)	7 (11.67)	8 (13.33)		
Cure	105 (87.50)	53 (88.33)	52 (86.67)		

**Table 3:** Comparison of pain scores between the two groups.

	*N*	1 day after operation	3 days after operation	Difference	*t*	*p*
Observation group	60	3.88 ± 0.90	1.83 ± 0.74	−2.05 ± 1.08	14.700	<0.001
Experimental group	60	3.75 ± 0.89	1.22 ± 0.67	−2.53 ± 0.96	20.336	<0.001

**Table 4:** Comparison of KSS clinical scores in different time periods.

	Preoperative KSS	KSS 1 day after operation	KSS 3 days after operation	KSS after 1 month	*F*	*p*
Observation group	48.92 ± 6.29d	50.58 ± 6.16c	69.77 ± 3.81b	87.40 ± 2.43a	997.099	<0.001
Experimental group	48.90 ± 5.34d	51.52 ± 6.36c	76.67 ± 5.20b 76.67	91.97 ± 2.3 a	1194.296	<0.001
*F*	0.000	0.667	68.734	111.462		
*p*	0.988	0.416	<0.001	<0.001		

Intergroup effects	*F* = 30.524, *pF* = 0.001					
Intragroup effects	*F* = 2184.398, *pF* = 0.001					
Intergroup*∗*intragroup	*F* = 15.004, *pF* = 0.001					

## Data Availability

The data used to support the findings of this study are available from the corresponding author (18650358018zyl@fjmu.edu.cn) upon request.
